The article "To Explore and Analyze the Safety and Clinical Efficacy of Periocline-Assisted Periodontal Basic Therapy on Chronic Periodontitis" was retracted in 2023. Reasons: unreliable results or conclusions; concerns about the data; concerns about the peer review; concerns about the citations.

# To Explore and Analyze the Safety and Clinical Efficacy of Periocline-Assisted Periodontal Basic Therapy on Chronic Periodontitis

**DOI:** 10.1155/2022/4601259

**Published:** 2022-09-12

**Authors:** Shengnan Zhang, Hongyan Ye, Jing Sun, Dongdong Tong, Junru Meng

**Affiliations:** ^1^Jinan Stomatological Hospital East Branch, Jinan Stomatological Hospital, Jinan, China; ^2^Department of Periodontology, Jinan Stomatological Hospital, Jinan, China; ^3^Department of Oral and Maxillofacial Surgery, School and Hospital of Stomatology, Cheeloo College of Medicine, Shandong University & Shandong Key Laboratory of Oral Tissue Regeneration & Shandong Engineering Laboratory for Dental Materials and Oral Tissue Regeneration, Jinan, China; ^4^Hospital Infection Management Office, Jinan Stomatological Hospital, Jinan, China

## Abstract

**Objective:**

This study aimed to investigate and analyse the clinical efficacy and safety of periocline-assisted periodontal foundation in the therapy of chronic periodontitis.

**Methods:**

From May 2018 to January 2021, 108 patients with chronic periodontitis were treated at our institution and randomly assigned equally to either the control or the experimental group. The plaque index (PLI), sulcus bleeding index (SBI), probing depth (PD), and periodontal attachment level (AI) were evaluated before and after periodontal basic therapy in the control group and periocline as an adjunct in the experimental group. Lactobacillus (LB) and *Porphyromonas gingivalis* (PG) concentrations in saliva were measured before and after therapy, and adverse responses during treatment were noted.

**Results:**

The levels of PLI, SBI, PD, and AI in the two groups were significantly lower in both groups at 1 and 3 months posttreatment compared to baseline; the levels of PLI and SBI were higher, and the levels of PD and AI were lower at 3 months after treatment compared to 1 month after treatment; compared with the control group at 1 month and 3 months after treatment, the levels of PLI, SBI, PD, and AI in the experimental group were lower than those in the control group (*P* < 0.05). The LB level was higher and the PG level was lower in both groups compared to baseline at 1 and 3 months posttreatment. The LB level was higher and the PG level was lower at 3 months posttreatment compared to 1 month after treatment. Compared with the control group at 1 month and 3 months after treatment, the LB level was higher, and the PG level was lower in the experimental group (*P* < 0.05). No significant adverse effects were observed in either group during the treatment period. Only 1 patient in the experimental group had mild gastrointestinal reactions, mainly nausea, without obvious neurological symptoms or abnormal blood changes, which did not affect the treatment.

The article "To Explore and Analyze the Safety and Clinical Efficacy of Periocline-Assisted Periodontal Basic Therapy on Chronic Periodontitis" was retracted in 2023. Reasons: unreliable results or conclusions; concerns about the data; concerns about the peer review; concerns about the citations.

**Conclusion:**

Periodontal fundamental therapy with perioclines may be a potential treatment for persistent periodontitis. It improves the primary clinical indicators, increases dysbacteriosis control, and has a strong safety profile. It could effectively control the development of clinical symptoms of periodontitis and reduce tissue destruction, with obvious clinical treatment effects. It could be used as the first choice for topical treatment of chronic periodontitis. It is recommended for further study by a wide range of researchers.

## 1. Introduction

As one of the most common periodontal diseases, the development of chronic periodontitis is closely related to the presence of plaque biofilm, an inflammatory disease with extensive involvement of periodontal supporting tissues, which could lead to tooth loss as well as systemic inflammation and is a major cause of tooth loss in adults [1]. According to the Guinness World Records, periodontal disease is the most common human disease and severe periodontitis is the sixth most prevalent disease in the world with an overall prevalence of 11.2% [2]. Globally, the loss of productivity due to severe periodontitis is estimated at 54 billion dollars per year. A number of complex microorganisms such as *Bacillus coelicolor*, *Porphyromonas gingivalis*, dense spirochetes of dental tartar, and actinomycetes are the most important pathogens causing periodontal disease. The main goal of periodontal treatment is plaque control and microbial reduction, and the main treatment measures include mechanical debridement and the use of topical and systemic antibiotics [3]. Although antibiotics could reduce periodontal pathogens, their frequent use could also lead to the development of bacterial resistance problems, in addition to gastrointestinal reactions, drug allergies, and periodontal pockets that have not reached the appropriate drug concentration. Scaling and root surface planning (SRP) is the most common treatment modality for most chronic periodontitis, but there are still limitations, such as the complex anatomical morphology of the root bifurcation, the depth of the periodontal pocket, and the deep penetration of microorganisms into the tissue making the removal of periodontal pathogenic bacteria particularly difficult, hence the importance of finding effective adjunctive treatment modalities for the treatment of chronic periodontitis [4, 5].

As a local sustained-release drug used to treat the disease in recent years, periocline is a broad-spectrum antibiotic with significant efficacy against tetracycline-sensitive or -resistant *Staphylococcus aureus*. The main ingredient of periocline ointment is minocycline hydrochloride, which has a broad-spectrum and highly effective antibacterial action. It prevents the synthesis of proteins from periodontitis pathogenic bacteria, promotes the regeneration of periodontal membrane cells, and facilitates the formation of new periodontal attachments. As a new periodontal slow-release drug, it has gradually been accepted by dentists, but its efficacy has been reported to vary in clinical work [6].

The article "To Explore and Analyze the Safety and Clinical Efficacy of Periocline-Assisted Periodontal Basic Therapy on Chronic Periodontitis" was retracted in 2023. Reasons: unreliable results or conclusions; concerns about the data; concerns about the peer review; concerns about the citations.

Our hospital has attempted to use periocline in addition to the routine periodontal basic treatment to treat periodontitis. The results are as follows.

## 2. Materials and Methods

### 2.1. General Data

A total of 108 patients with chronic periodontitis who were treated in our hospital from May 2018 to January 2021 were selected and evenly randomized into the control group and experimental group. There were 30 males and 24 females in the control group, age ranging from 23 to 64 years, with an average of 41.26 ± 4.12 years.

The randomization was carried out using an online web-based randomization tool (freely available at http://www.randomizer.org/). For concealment of allocation, the randomization procedure and assignment were managed by an independent research assistant who was not involved in screening or evaluation of the participants.

The original sample size calculation estimated that 50 patients in each group would be needed to detect a 3-point difference between groups in a 2-sided significance test with a power of 0.8 and an alpha error level of 0.05.

The study protocol and all amendments were approved by the appropriate ethics committee at each centre. The study was done in accordance with the protocol, its amendments, and standards of Good Clinical Practice. All participants provided written informed consent before enrolment. The study was reviewed and approved by the ethics committee of our hospital (approval no. 297917-197).

There were 32 males and 22 females in the experimental group, aged from 21 to 65 years, with an average of 41.10 ± 4.25 years. The baseline data were balanced in the two groups, and they were comparable.

### 2.2. Inclusion and Exclusion Criteria

#### 2.2.1. Inclusion Criteria

1. All were diagnosed after examination in our hospital
2. Patients with more than 10 remaining teeth in the oral cavity, at least 2 teeth with probing depth (PD) ≥6 mm, and attachment loss of >5 mm
3. Patients who had not received periodontal treatment in the past 1 year and had not been treated with antibiotics one month prior to commencing recruitment
4. Patients with no previous history of tetracycline allergy

The article "To Explore and Analyze the Safety and Clinical Efficacy of Periocline-Assisted Periodontal Basic Therapy on Chronic Periodontitis" was retracted in 2023. Reasons: unreliable results or conclusions; concerns about the data; concerns about the peer review; concerns about the citations.

#### 2.2.2. Exclusion Criteria

1. Patients with systemic diseases and who are breastfeeding and pregnant
2. Patients with pulp inflammation and who are unable to come to the hospital in time for follow-up
3. Patients with systemic diseases such as diabetes and cardiovascular disease, where it is anticipated that the associated disease may affect the development of CP and the efficacy of periodontal treatment
4. Patients who have taken medications such as antibiotics before and after treatment that may affect periodontal tissues or the efficacy of treatment
5. Patients with systemic diseases such as diabetes and cardiovascular disease, where it is anticipated that the associated disease may affect the development of CP and the efficacy of periodontal treatment
6. Patients who have taken medications such as antibiotics before and after treatment that may affect periodontal tissues or the efficacy of treatment
7. Patients with aggressive periodontitis and other types of periodontitis, patients who have received other periodontal treatment within 6 months, and women during pregnancy

### 2.3. Methods

Both groups were offered basic periodontal treatment, including full-mouth supragingival scaling, with a follow-up visit conducted one week after supragingival scaling. After measuring the tooth index, a rinse with 3% hydrogen peroxide was applied after subgingival scaling and root planing [7].

In the experimental group, periocline treatment was additionally treated as follows: The periocline ointment was gently injected into the patient's periodontal pocket to the bottom of the pocket until the ointment is able to spill out of the periodontal pocket. Patients were instructed to refrain from eating and gargling within 2 hours after administered. The drug is administered once a week for consecutive 4 weeks of treatment. The control group was treated with iodine glycerine, and the frequency and duration of treatment were the same as in the experimental group.

### 2.4. Efficacy Evaluation Criteria

The plaque index (PLI), sulcus bleeding index (SBI), PD, and periodontal attachment level (AI) of the two groups before treatment, 1 month, and 3 months after treatment were compared. The concentrations of Lactobacillus (LB) and *Porphyromonas gingivalis* (PG) in saliva were compared between the two groups before and after treatment, and adverse reactions during treatment were observed.

### 2.5. Statistical Analysis

If the parameter beta is either a difference of means, a log odds ratio, or a log hazard ratio, then it is reasonable to assume that *b* is unbiased and normally distributed. All statistical analyses were performed using SPSS18.0 statistical software. Measurement data were expressed as mean ± standard deviation (*x*±*s*), and the differences between groups were compared using one-way ANOVA followed by Student's *t* test. Statistical significance was set at *P* < 0.05.

The article "To Explore and Analyze the Safety and Clinical Efficacy of Periocline-Assisted Periodontal Basic Therapy on Chronic Periodontitis" was retracted in 2023. Reasons: unreliable results or conclusions; concerns about the data; concerns about the peer review; concerns about the citations.

## 3. Results

### 3.1. Comparison of PLI, SBI, PD, and AI between the Two Groups before Treatment, 1 Month, and 3 Months after Treatment

There was no statistically significant difference in the levels of PLI, SBI, PD, and AI between the two groups before treatment (*P* > 0.05). At 1 month and 3 months after treatment, the levels of PLI, SBI, PD, and AI in the two groups decreased significantly from baseline after treatment; PLI and SBI levels were higher and PD and AI levels at 3 months posttreatment were lower compared to 1 month posttreatment; the levels of PLI, SBI, PD, and AI in the experimental group were lower than those in the control group at 1 month and 3 months after treatment (*P* < 0.05) (Table 1).

### 3.2. Comparison of LB and PG between the Two Groups before Treatment, 1 Month, and 3 Months after Treatment

The difference in LB and PG levels between the two groups before treatment was not statistically significant (*P* > 0.05). The LB level was greater and the PG level was decreased in both groups at 1 month and 3 months after treatment. LB levels increased and PG levels decreased after 3 months compared to 1 month after treatment. At 1 month and 3 months following treatment, the experimental group had greater LB levels and lower PG levels than the control group (*P* < 0.05) (Table 2).

### 3.3. Comparison of Adverse Reactions between the Two Groups

No significant adverse reactions occurred during treatment in either group. Only one patient in the experimental group experienced mild gastrointestinal reactions, mainly nausea, without obvious neurological symptoms or abnormal blood changes, which did not affect the treatment.

## 4. Discussion

Periodontitis is a chronic infectious disease that occurs in the supporting tissues of the periodontium and is a complex multifactorial disease characterised by the destruction of periodontal connective tissue and the loss of alveolar bone, which is one of the most common diseases in the clinical oral cavity and the most significant cause of tooth loss in humans. Periodontal tissue destruction is a process in which oral bacterial infection acts as an initiating factor, thereby inducing early inflammation [8, 9]. During the developmental phase of the disease, anaerobic bacteria predominate, with *Porphyromonas gingivalis*, *Proteus intermedius*, and *Clostridium perfringens* being the main bacteria involved. At the same time, after the disease has progressed, parthenogenic anaerobes are also involved, mainly *Streptococcus pyogenes*, *Staphylococcus aureus*, and *Staphylococcus epidermidis*. These microorganisms could produce and release proteolytic enzymes and toxic metabolites that cause damage to periodontal tissues, and factors related to inflammation could also be produced through their stimulation of host cells [10, 11]. Therefore, in recent years, with the development of preventive dentistry, oral bacteria, soft tartar, and tartar have become the main target of prevention and treatment, but only with periodontal mechanical and surgical treatment can not completely control the inflammation around them. Some of the periodontal pathogenic bacteria are found deep in the soft tissues and dentin layers of the periodontium as well as in areas that cannot be reached by surgical instruments; therefore, pharmacological treatment can play an adjunctive role in basic periodontal treatment as well as surgical treatment [12, 13].

The article "To Explore and Analyze the Safety and Clinical Efficacy of Periocline-Assisted Periodontal Basic Therapy on Chronic Periodontitis" was retracted in 2023. Reasons: unreliable results or conclusions; concerns about the data; concerns about the peer review; concerns about the citations.

At present, the most commonly used basic periodontal treatments are scaling, subgingival scaling, and root planning. With the exception of some patients with severe periodontitis, other degrees of periodontitis require basic treatment to achieve satisfactory clinical results. The report pointed out the remarkable success of pharmacological treatment as a common adjunct to periodontal disease. Periocline is an ointment with 2% minocycline as the main ingredient in an extended release ointment that is widely used and easily absorbed. During application, the ointment could be penetrated into the skin using a needle. Deep periodontal pocket ensures that plasma concentration could be maintained in the deep periodontal pocket for a long time [14, 15].

At the same time, pharmacological tests have shown that the application of periocline is effective in killing periodontal pathogens such as porphyromonas gingivalis and aggregate actinobacteria; moreover, the bactericidal effect lasts for a long time. In addition, it is relatively easy to operate and is considered to be the most commonly used periodontal pocket drug in current clinical work [16, 17]. A comprehensive review has shown that previous studies indicated that topical adjuvant therapy with periocline on the basis of traditional periodontal treatment had greater curative outcomes and reduced periodontal disease symptoms in patients [18, 19].

In this study, our hospital observed the clinical efficacy and safety of periocline-assisted periodontal basic therapy on chronic periodontitis. The levels of PLI, SBI, PD, and AI were lower in the experimental group at 1 month and 3 months after therapy than in the control group. This is thought to be because periocline has a strong inhibitory effect on collagenase activity associated with periodontal destruction, effectively preventing and arresting periodontal tissue damage, promoting root surface decalcification and migration of connective tissue over the root, and accelerating the formation of new periodontal attachments [20]. As a topical slow-release drug, dimethyltetracycline hydrochloride is the main component of periocline ointment, which could effectively kill anaerobic bacteria and parthenogenic anaerobic bacteria. It could be slowly released in the periodontal pockets of patients with chronic periodontitis to maintain effective local antibacterial and bactericidal concentrations, and there are still high antibacterial and bactericidal concentrations in the periodontal pockets of patients within 5–7 days of administration, which can inhibit alveolar bone resorption, enhance the regenerative function of periodontal tissues, and prompt the stimulation of periodontal membrane by exposed collagen and its continuous migration on the root surface, thus directly accelerating cell attachment and growth [21].

The article "To Explore and Analyze the Safety and Clinical Efficacy of Periocline-Assisted Periodontal Basic Therapy on Chronic Periodontitis" was retracted in 2023. Reasons: unreliable results or conclusions; concerns about the data; concerns about the peer review; concerns about the citations.

Additionally, studies have reported the presence of a large number of microorganisms in the normal oral environment. These microorganisms depend on the surrounding environment for growth and reproduction and furthermore maintain a dynamic dependence and mutual restriction relationship with the organism [22, 23]. When periodontal disease arises, the oral flora alters, manifesting as low levels of LB and a high levels of PG. The results indicated that after the addition of periocline, the experimental group had a higher LB level and lower PG level than the control group at 1 month and 3 months after treatment. This would imply that periocline adjunctive therapy could successfully combat periodontal infections while also substantially improving the efficacy of standard periodontal treatment [24]. Periocline is a broad-spectrum antibiotic with a potent inhibitory effect on a range of periodontal pathogens, mainly *Porphyromonas gingivalis*, and is more convenient as a topical extended-release drug that is administered via a single injectable syringe directly to the base of the periodontal pocket and does not require multiple doses. The drug could prevent or reduce plaque production, promote rapid healing of the heel cusps, and facilitate the repair of periodontal tissue [25].

However, this study has a number of shortcomings due to a number of constraints: (1) In terms of the study sample, the sample size ultimately collected for this trial was relatively small and did not allow for a more comprehensive and objective evaluation of the significant differences in efficacy between the two treatment groups from a large sample size perspective. (2) In terms of observational indicators and efficacy, this study used a large number of subjective efficacy criteria, and it is difficult to give an absolutely objective and accurate description of the scale because of the wide variation in subjective perceptions between individuals, their different levels of education, and their understanding of the questions on the scale. (3) In terms of follow-up time, the short follow-up period after treatment in this trial did not allow for a better observation of the long-term treatment effects.

The article "To Explore and Analyze the Safety and Clinical Efficacy of Periocline-Assisted Periodontal Basic Therapy on Chronic Periodontitis" was retracted in 2023. Reasons: unreliable results or conclusions; concerns about the data; concerns about the peer review; concerns about the citations.

## 5. Conclusion

To sum up, periocline-assisted periodontal basic therapy is a highly promising solution for chronic periodontitis. It improves the major clinical indicators and promotes the regulation of dysbacteriosis, with a high safety profile. Ongoing studies with a larger sample size and more observation indicators are necessary to further validate the benefits of periocline-assisted therapy.

## Figures and Tables

**Table 1:** Comparison of PLI, SBI, PD, and AI between the two groups before treatment, 1 month, and 3 months after treatment.

Groups	Timing	PLI	SBI	PD	AI
Control group	Before treatment	1.35 ± 0.51	4.29 ± 1.15	7.31 ± 0.65	7.41 ± 0.95
	One month after treatment	0.83 ± 0.34	2.69 ± 1.30	6.11 ± 0.73	6.36 ± 0.91
	Three months after treatment	1.54 ± 0.48	2.72 ± 1.29	0.45 ± 0.79	5.45 ± 0.85
*F*		6.214	4.251	6.258	7.115
*P*		0.01	0.001	0.001	0.001

Experimental group	Before treatment	1.35 ± 0.53	4.32 ± 1.16	7.29 ± 0.65	7.43 ± 0.90
	One month after treatment	0.74 ± 0.39	1.95 ± 0.91	5.50 ± 0.64	5.83 ± 0.88
	Three months after treatment	1.12 ± 0.36	2.35 ± 1.36	4.31 ± 0.68	4.75 ± 0.90
*F*		16.587	12.258	10.987	13.687
*P*		≤0.001	≤0.001	≤0.001	≤0.001

**Table 2:** Comparison of LB and PG between the two groups before treatment, 1 month, and 3 months after treatment.

Groups	Timing	LB (CFU/ml, 1 × 10^6^)	PG (CFU/ml, 1 × 10^6^)
Control group	Before treatment	0.05 ± 0.02	3.24 ± 1.04
	One month after treatment	2.95 ± 1.62	2.98 ± 0.68
	Three months after treatment	5.32 ± 1.55	2.41 ± 0.55
*F*		6.574	8.110
*P*		0.001	0.001

Experimental group	Before treatment	0.06 ± 0.01	3.26 ± 1.11
	One month after treatment	4.12 ± 1.58	2.43 ± 0.71
	Three months after treatment	6.46 ± 0.61	1.68 ± 0.23
*F*		19.544	1.226
*P*		≤0.001	≤0.001

## Data Availability

All data generated or analysed during this study are included in this published article.
